The article "RBFNN-Based Singularity-Free Terminal Sliding Mode Control for Uncertain Quadrotor UAVs" was published in 2021. Journal: Comput Intell Neurosci.

# RBFNN-Based Singularity-Free Terminal Sliding Mode Control for Uncertain Quadrotor UAVs

**DOI:** 10.1155/2021/3576783

**Published:** 2021-08-19

**Authors:** Meiling Tao, Xiongxiong He, Shuzong Xie, Qiang Chen

**Affiliations:** ^1^Data-driven Intelligent Systems Laboratory, College of Information Engineering, Zhejiang University of Technology, Hangzhou 310023, China; ^2^Key Laboratory of Advanced Perception and Intelligent Control of High-end Equipment, Ministry of Education, Anhui Polytechnic University, Wuhu 241000, Anhui Province, China

## Abstract

In this article, a singularity-free terminal sliding mode (SFTSM) control scheme based on the radial basis function neural network (RBFNN) is proposed for the quadrotor unmanned aerial vehicles (QUAVs) under the presence of inertia uncertainties and external disturbances. Firstly, a singularity-free terminal sliding mode surface (SFTSMS) is constructed to achieve the finite-time convergence without any piecewise continuous function. Then, the adaptive finite-time control is designed with an auxiliary function to avoid the singularity in the error-related inverse matrix. Moreover, the RBFNN and extended state observer (ESO) are introduced to estimate the unknown disturbances, respectively, such that prior knowledge on system model uncertainties is not required for designing attitude controllers. Finally, the attitude and angular velocity errors are finite-time uniformly ultimately bounded (FTUUB), and numerical simulations illustrated the satisfactory performance of the designed control scheme.

## 1. Introduction

Due to the advantages of a large range of applications of QUAVs, the attitude control of QUAVs has received extensive attention in many fields. Designing a suitable control law according to the type of flight mission is important for the study of QUAVs attitude control [1]. However, the control scheme proposed in [1] only achieves the asymptotic convergence of the attitude or tracking error, which means that the system states converge to zero within an infinite time. In practical applications, the controller design needs specific requirements for convergence speed and control accuracy. Thus, finite-time control (FTC) methods have been proposed to deal with the control problems of different nonlinear systems [2–4]. In [2], a parameter update law was constructed to compensate for parameter uncertainty, and an adaptive sliding mode control (SMC) scheme was constructed to ensure the finite-time convergence of the tracking error of QUAV. In [3], combining integral backstepping technology and terminal SMC, a FTC method was designed to guarantee the position and attitude tracking stability of QUAVs, such that the system states are semiglobal practical FTUUB. In [4], a FTC scheme was proposed to guarantee the finite-time convergence of position and attitude states in the QUAV tracking error system.

To solve the dependence of the FTC on a nonlinear system model, multiple control methods have the capability to approximate nonlinear functions, which is used to implement the estimation task of the nonlinear system, i.e., adaptive control [5] and optimal control [6]. In the past years, a method called RBFNN has been widely introduced to approximate the dynamic parameters of nonlinear systems, such that no prior knowledge of model information is required in [7, 8]. In [7], a RBFNN method was devolved to estimate the unknown model uncertainties of robot manipulators. In [8], a RBFNN-based SMC scheme was presented to guarantee the asymptotic convergence of the system states under the model uncertainties. Compared with other estimation methods [5, 6], RBFNN has faster convergence speed and local approximation capability to avoid local minima problems. Thus, RBFNN is more suitable for real-time control, such as QUAV attitude control.

Moreover, for complex coupled systems, extended state observer (ESO) as an alternative approach to solve the bounded disturbances is used to decouple the system by treating the coupling terms as a part of the lumped uncertainties. Due to its satisfactory disturbance estimation, ESO-based controllers are widely applied in different practical nonlinear systems, such as rigid spacecrafts [9] and robot manipulators [10]. In [9], a SMC based on backstepping and ESO methods was used to achieve a faster convergence in the rigid spacecraft attitude control system. In [10], an FTC with the model-assisted ESO was used to compensate the bounded uncertainties and guarantee the finite-time convergence of the system states. Although RBFNN and ESO have been successfully applied to a variety of uncertain nonlinear systems [7–10], it is less used in QUAVs.

Inspired by the above discussions, an RBFNN-based finite-time adaptive attitude tracking controller is designed for the attitude tracking problem of QUAVs with inertial uncertainty and unknown external disturbances, and the main contributions are summarized in the following:

- Instead of employing any piecewise continuous functions, a SFTSMS is proposed to avoid the singularity directly in the differential of the sliding variable
- An auxiliary function is designed to handle a potential singularity resulted from the use of the error-related inverse matrix in the attitude controller design
- By employing RBFNN and ESO to estimate the unknown dynamics, prior knowledge on system model uncertainties is not required in the controller design, and the tracking errors are FTUUB by the proposed control law

The structure of this article is given as follows. The attitude model and necessary preliminaries are given in Section 2.  Section 3 shows the detailed design process of SFTSMS. Controller design and rigorous theoretical proofs are depicted in Sections 4 and 5, respectively.  Section 6 shows the effective simulations, and the conclusion is given in Section 7.

## 2. Model Description and Preliminaries

### 2.1. Quadrotor Attitude Dynamics

As depicted in Figure 1, the dynamics of the QUAV is represented as follows [11]:

(1) $$\begin{array}{c} {\dot{q}}_{0}=-\frac{1}{2}q_{v}^{T}\omega ,\\ {\dot{q}}_{v}=\frac{1}{2}\left(q_{v}^{\times }+q_{0}I_{3}\right)\omega , \end{array}$$

where *q*_0_ ∈ *R* and *q*_*v*_=[*q*_1_, *q*_2_, *q*_3_]^*T*^ ∈ *R*^3×1^ denote the scalar and vector elements of the unit quaternion *Q*=[*q*_0_, *q*_*v*_^*T*^]^*T*^, respectively, and *I*_3_ ∈ *R*^3×3^ is the identity matrix, and the skew-symmetric matrix *A*^×^ ∈ *R*^3×3^ is given by

(2) $$\begin{array}{c} A^{\times }=\left[\begin{array}{ccc} 0 & -A_{3} & A_{2}\\ A_{3} & 0 & -A_{1}\\ -A_{2} & A_{1} & 0 \end{array}\right]. \end{array}$$

The reference attitude vector is defined as *Q*^*r*^=[*q*_0_^*r*^, *q*_1_^*r*^, *q*_2_^*r*^, *q*_3_^*r*^]^*T*^ ∈ *R*^4×1^, and ${\dot{Q}}^{r}$ and ${\ddot{Q}}^{r}$ are bounded. The attitude tracking error *e*_*q*_ is

(3) $$\begin{array}{c} e_{q}=E\left(Q^{r},Q\right)=2\left(q_{0}^{r}q_{0}+\sum_{i=1}^{3}q_{i}^{r}q_{i}\right)\times \left[\begin{array}{c} -q_{0}^{r}q_{1}+q_{1}^{r}q_{0}+q_{2}^{r}q_{3}-q_{3}^{r}q_{2}\\ -q_{0}^{r}q_{2}-q_{1}^{r}q_{3}+q_{2}^{r}q_{0}+q_{3}^{r}q_{1}\\ -q_{0}^{r}q_{3}+q_{1}^{r}q_{2}-q_{2}^{r}q_{2}+q_{3}^{r}q_{0} \end{array}\right], \end{array}$$

and the dynamics model is expressed as

(4) $$\begin{array}{c} J\dot{\omega }=-\omega^{\times }J\omega +u+d, \end{array}$$

where *ω* ∈ *R*^3×1^ denotes the angular velocity, *J* ∈ *R*^3×3^ is a positive definite inertia matrix, *u*=[*u*_1_, *u*_2_, *u*_3_]^*T*^ ∈ *R*^3×1^ represents the generalized control torque produced by rotating propellers, and *d*=[*d*_1_, *d*_2_, *d*_3_]^*T*^ ∈ *R*^3×1^ denotes the unknown but bounded continuous external disturbances.

Defining *J*=*J*_0_+Δ*J*, (4) is expressed as

(5) $$\begin{array}{c} J_{0}\dot{\omega }=-\omega^{\times }J_{0}\omega -\omega^{\times }\Delta J\omega -\Delta J\dot{\omega }+u+d, \end{array}$$

where *J*_0_ and Δ*J* are denoted as the nominal and the unknown inertia matrix, respectively.

The angular velocity tracking error is

(6) $$\begin{array}{c} e_{\omega }=\omega -\omega^{r}, \end{array}$$

where *ω*^*r*^ is given by

(7) $$\begin{array}{c} \omega^{r}=2\left[\begin{array}{c} -q_{2}^{r}{\dot{q}}_{v1}^{r}+q_{0}^{r}{\dot{q}}_{v1}^{r}+q_{v3}^{r}{\dot{q}}_{v2}^{r}-q_{v2}^{r}{\dot{q}}_{v3}^{r}\\ -q_{v2}^{r}{\dot{q}}_{0}^{r}-q_{v3}^{r}{\dot{q}}_{v1}^{r}+q_{0}^{r}{\dot{q}}_{v2}^{r}+q_{v1}^{r}{\dot{q}}_{v3}^{r}\\ -q_{v3}^{r}{\dot{q}}_{0}^{r}+q_{v2}^{r}{\dot{q}}_{v1}^{r}-q_{v1}^{r}{\dot{q}}_{v2}^{r}+q_{0}^{r}{\dot{q}}_{v3}^{r} \end{array}\right]. \end{array}$$

From (5)–(7), the tracking error model is expressed as

(8) $$\begin{array}{c} {\dot{e}}_{q}=e_{\omega },\\ {\dot{e}}_{\omega }=-J_{0}^{-1}\omega^{\times }J_{0}\omega -J_{0}^{-1}\omega^{\times }\Delta J\omega -J_{0}^{-1}\Delta J\dot{\omega }+J_{0}^{-1}u+J_{0}^{-1}d-{\dot{\omega }}^{r}. \end{array}$$

**Remark 1 .**

Unit quaternion is able to represent the attitude uniquely because the equilibrium states correspond to a unique physical equilibrium orientation [12] in the QUAV.

### 2.2. RBFNN

In practical systems, neural networks (NNs) are online estimation techniques for unknown nonlinear uncertainties. Due to the approximation characteristics and faster learning convergence, RBFNN is widely used in the estimation of nonlinear functions in the field of control. This section will introduce the structure of RBFNN.

RBFNN consists of three parts: input layer, output layer, and hidden layer. As shown in Figure 2, *x* ∈ [*x*_1_, *x*_2_,…,*x*_*n*_]^*T*^ is the neural network input vector, *W* ∈ [*W*_1_, *W*_2_,…,*W*_*m*_]^*T*^ is the weight of the *m*th network node, *y* represents the output vector, and *ϕ*(*x*)=[*ϕ*_1_, *ϕ*_2_,…,*ϕ*_*m*_]^*T*^ is the basis function, which can approximate nonlinear uncertainties with high precision through the linear combination of Gaussian functions, which is given by the following [7]:

(9) $$\begin{array}{c} \phi_{k}\left(x\right)=\exp\left[\frac{-{\left(x-\mu_{k}\right)}^{T}\left(x-\mu_{k}\right)}{a_{k}^{2}}\right],\;k=1,2,\ldots ,m, \end{array}$$

where *μ*_*k*_ is the center of the RBF and *a*_*k*_ means the scaling parameter of the network node *m*.

Thus, the output vector *y* is expressed as

(10) $$\begin{array}{c} y=\sum_{k=1}^{m}W_{k}\phi_{k}. \end{array}$$

Considering that RBFNN has good nonlinear approximation ability [13], the approximate system model of the nonlinear function *F* is

(11) $$\begin{array}{c} F\left(x\right)=W^{T}\phi \left(x\right)+\varepsilon , \end{array}$$

where *ε* represents the estimation error.

### 2.3. Useful Lemmas

**Lemma 1 (see [14]).**

For Λ_1_ > 0, Λ_2_ > 0, and 0 < *ι* < 1, a Lyapunov condition of finite-time stability is expressed as $\dot{V}\left(x\right)+\Lambda_{1}V\left(x\right)+\Lambda_{2}V^{\iota }\left(x\right)\leq 0$, where the settling time satisfies *T*_0_ ≤ (1/Λ_1_(1 − *ι*))ln(Λ_1_*V*^1−*ι*^(*x*_0_)+Λ_2_/Λ_2_), where *V*(*x*_0_) represents the initial state of *V*(*x*).

**Lemma 2 (see [15]).**

Given *a*_1_, *a*_2_,…, *a*_*n*_ > 0 and *p* > 0, the following relationships hold:

(12) $$\begin{array}{c} \left\{\begin{array}{cc} \sum_{i=1}^{n}a_{i}^{p}\geq n^{1-p}{\left(\sum_{i=1}^{n}a_{i}\right)}^{p}, & p>1,\\ \sum_{i=1}^{n}a_{i}^{p}\geq {\left(\sum_{i=1}^{n}a_{i}\right)}^{p}, & 0<p<1. \end{array}\right. \end{array}$$

**Lemma 3 (see [16]).**

Given a continuous function *f*(*x*)=*x*^*ι*^ − *ιx* with 1 ≤ *ι* ≤ 2, for any *x* > 0, there exists the following inequality:

(13) $$\begin{array}{c} \frac{x^{\iota }}{\iota }\geq x+\frac{1-\iota }{\iota }. \end{array}$$

## 3. SFTSMS and Auxiliary Function Design

### 3.1. SFTSMS

A SFTSMS is constructed as

(14) $$\begin{array}{c} S=\text{sig}\left(e_{q}\right)+\frac{\Lambda_{1}}{2-a}{\text{sig}}^{2-a}\left(e_{\omega }+\Lambda_{2}\text{sig}\left(e_{q}\right)\right), \end{array}$$

where *S*=[*S*_1_, *S*_2_, *S*_3_]^*T*^ ∈ *R*^3×1^, Λ_1_ > 0, Λ_2_ > 0, and 0 < *a*=*a*_1_/*a*_2_ < 1, *a*_1_ and *a*_2_ are positive odd integers, and the term sig^*r*^(*x*) is given by

(15) $$\begin{array}{c} {\text{sig}}^{r}\left(x\right)={\left[{\left|x_{1}\right|}^{r}\mathrm{sgn}\left(x_{1}\right),{\left|x_{2}\right|}^{r}\mathrm{sgn}\left(x_{2}\right),{\left|x_{3}\right|}^{r}\mathrm{sgn}\left(x_{3}\right)\right]}^{T}, \end{array}$$

where *x*=[*x*_1_, *x*_2_, *x*_3_]^*T*^*R*^3×1^ and *r* > 0.

The time derivative of (14) is expressed as

(16) $$\begin{array}{c} \dot{S}=e_{\omega }+\Lambda_{1}{\left|e_{\omega }+\Lambda_{2}\text{sig}\left(e_{q}\right)\right|}^{1-a}\cdot \left({\dot{e}}_{\omega }+\Lambda_{2}e_{\omega }\right). \end{array}$$

Due to the facts that 1 − *a* > 0, the singularity will not occur in (16).

When *S*=0, (14) is rewritten as

(17) $$\begin{array}{c} \text{sig}\left(e_{q}\right)+\frac{\Lambda_{1}}{2-a}{\text{sig}}^{2-a}\left(e_{\omega }+\Lambda_{2}\text{sig}\left(e_{q}\right)\right)=0. \end{array}$$

According to 2 − *a* > 1, the following equation is obtained as

(18) $$\begin{array}{c} {\left(\frac{2-a}{\Lambda_{1}}\right)}^{1/2-a}{\text{sig}}^{1/2-a}\left(e_{q}\right)=-\left(e_{\omega }+\Lambda_{2}\text{sig}\left(e_{q}\right)\right). \end{array}$$

From (18), the equivalent equation of (14) is obtained as follows [12]:

(19) $$\begin{array}{c} s=e_{\omega }+\Lambda_{2}\text{sig}\left(e_{q}\right)+{\left(\frac{2-a}{\Lambda_{1}}\right)}^{1/2-a}{\text{sig}}^{1/2-a}\left(e_{q}\right)=0. \end{array}$$

From (8) and (19), one has

(20) $$\begin{array}{c} {\dot{e}}_{q}=-\Lambda_{2}\text{sig}\left(e_{q}\right)-{\left(\frac{2-a}{\Lambda_{1}}\right)}^{1/2-a}{\text{sig}}^{1/2-a}\left(e_{q}\right). \end{array}$$

To illustrate *e*_*q*_ is finite-time convergent, a Lyapunov function is chosen as

(21) $$\begin{array}{c} V_{1}=\frac{1}{2}e_{q}^{T}e_{q}. \end{array}$$

From (20), the time derivative of *V*_1_ is

(22) $$\begin{array}{c} {\dot{V}}_{1}=e_{q}^{T}{\dot{e}}_{q}=e_{q}^{T}\left[-\Lambda_{2}\text{sig}\left(e_{q}\right)-{\left(\frac{2-a}{\Lambda_{1}}\right)}^{1/2-a}{\text{sig}}^{1/2-a}\left(e_{q}\right)\right]\\ =-\Lambda_{2}{\left|e_{q}\right|}^{2}-{\left(\frac{2-a}{\Lambda_{1}}\right)}^{1/2-a}{\left|e_{q}\right|}^{1+\left(1/2-a\right)}=-{\bar{\Lambda }}_{1}V_{1}-{\bar{\Lambda }}_{2}V_{1}^{\iota_{0}}, \end{array}$$

where ${\bar{\Lambda }}_{1}=2\Lambda_{2}$, ${\bar{\Lambda }}_{2}=2^{3-a/4-2a}{\left(2-a/\Lambda_{1}\right)}^{1/2-a}$, and *ι*_0_=(1/2)+(1/4 − 2*a*).

According to Lemma 1 and (8), *e*_*q*_ and *e*_*ω*_ converge to the equilibrium within a finite-time *T*_*s*_ satisfying

(23) $$\begin{array}{c} T_{s}\leq \frac{1}{{\bar{\Lambda }}_{1}\left(1-\iota_{0}\right)}\ln\frac{{\bar{\Lambda }}_{1}V_{1}^{1-\iota_{0}}\left(e_{q}\left(0\right)\right)+{\bar{\Lambda }}_{2}}{{\bar{\Lambda }}_{2}}, \end{array}$$

where *e*_*q*_(0) represents the initial states of *e*_*q*_(*t*).

This completes the proof.

### 3.2. Auxiliary Function Design

Substituting (8) into (16) yields

(24) $$\begin{array}{c} \dot{S}=e_{\omega }+\Lambda_{1}{\left|e_{\omega }+\Lambda_{2}\text{sig}\left(e_{q}\right)\right|}^{1-a}\cdot \left(\begin{array}{c} -J_{0}^{-1}\omega^{\times }J_{0}\omega -J_{0}^{-1}\omega^{\times }\Delta J\omega -J_{0}^{-1}\Delta J\dot{\omega }\\ +J_{0}^{-1}Eu+D\left(t\right)-{\dot{\omega }}^{r}+\Lambda_{2}e_{\omega } \end{array}\right)\\ =e_{\omega }+Y\left(J_{0}^{-1}u+D-J_{0}^{-1}\omega^{\times }J_{0}\omega -J_{0}^{-1}\omega^{\times }\Delta J\omega -J_{0}^{-1}\Delta J\dot{\omega }-{\dot{\omega }}^{r}+\Lambda_{2}e_{\omega }\right)\\ =e_{\omega }+Y\left(F_{0}+D+J_{0}^{-1}u\right), \end{array}$$

where *Y*=diag(*Y*_1_, *Y*_2_, *Y*_3_) ∈ *R*^3×3^, *Y*_*i*_=Λ_1_|Θ_*i*_|^1−*a*^ with *i*=1,2,3, *e*_*q*_=[*e*_*q*1_, *e*_*q*2_, *e*_*q*3_]^*T*^, Θ=*e*_*ω*_+Λsig(*e*_*q*_), and $F_{0}=Y^{-1}\cdot e_{\omega }+D-J_{0}^{-1}\omega^{\times }J_{0}\omega -J_{0}^{-1}\omega^{\times }\Delta J\omega -J_{0}^{-1}\Delta J\dot{\omega }-{\dot{\omega }}^{r}+\Lambda_{2}e_{\omega }$.

Due to the existence of the term of *F*_0_ in the expression of *Y*^−1^, it may cause the potential singularity issue when Θ=0. Consequently, an auxiliary function *φ* is constructed to solve the singularity caused by *Y*^−1^ in the controller design.

Thus, (24) is expressed as

(25) $$\begin{array}{c} \dot{S}=Y\left(F_{0}+J_{0}^{-1}u\right)+e_{\omega }+\Lambda_{2}S-\Lambda_{2}S\\ =Y\left(J_{0}^{-1}u+D-J_{0}^{-1}\omega^{\times }J_{0}\omega -J_{0}^{-1}\omega^{\times }\Delta J\omega -J_{0}^{-1}\Delta J\dot{\omega }-{\dot{\omega }}_{r}\right)\\ +Y\cdot \Lambda_{2}e_{\omega }+\left(e_{\omega }+\Lambda_{2}S\right)-\Lambda_{2}S. \end{array}$$

From the definition of *S* and Θ, it has

(26) $$\begin{array}{c} e_{\omega }+\Lambda_{2}S=e_{\omega }+\Lambda_{2}\left(\text{sig}\left(e_{q}\right)+\frac{\Lambda_{1}}{2-a}{\text{sig}}^{2-a}\left(\Theta \right)\right)\\ =e_{\omega }+\Lambda_{2}\text{sig}\left(e_{q}\right)+\Lambda_{2}\cdot \frac{\Lambda_{1}}{2-a}{\text{sig}}^{2-a}\left(\Theta \right)=Y\cdot \left(\frac{1}{\Lambda_{1}}{\text{sig}}^{a}\left(\Theta \right)+\frac{\Lambda_{2}}{2-a}\Theta \right). \end{array}$$

From (26), the auxiliary function *φ* is defined as

(27) $$\begin{array}{c} \varphi =\frac{1}{\Lambda_{1}}{\text{sig}}^{a}\left(\Theta \right)+\frac{\Lambda_{2}}{2-a}\Theta , \end{array}$$

and (25) can be rewritten as

(28) $$\begin{array}{c} \dot{S}=ϒ\cdot \left(J_{0}^{-1}u+D-J_{0}^{-1}\omega^{\times }J_{0}\omega -J_{0}^{-1}\omega^{\times }\Delta J\omega -J_{0}^{-1}\Delta J\dot{\omega }-{\dot{\omega }}^{r}+\varphi +\Lambda_{2}e_{\omega }\right)\\ -\Lambda_{2}S=ϒ\left(J_{0}^{-1}u+F+D\right)-\Lambda_{2}S, \end{array}$$

where *F* denotes the lumped uncertainties presented by

(29) $$\begin{array}{c} F=-J_{0}^{-1}\omega^{\times }J_{0}\omega -J_{0}^{-1}\omega^{\times }\Delta J\omega -J_{0}^{-1}\Delta J\dot{\omega }-{\dot{\omega }}^{r}+\varphi +\Lambda_{2}e_{\omega }. \end{array}$$

## 4. Controller Design

### 4.1. ESO

The bounded external disturbances *D* in (28) are estimated by the ESO. Considering the disturbances *D* as an extended state, system (28) is rewritten as

(30) $$\begin{array}{c} \dot{S}=Y\left(J_{0}^{-1}u+D+F\right)-\Lambda_{2}S,\\ \dot{D}=h\left(t\right), \end{array}$$

where *h*(*t*) represents the derivative of *D*.

Then, the second-order ESO for (30) is constructed as

(31) $$\begin{array}{c} E_{1}=Z_{1}-S,\\ {\dot{Z}}_{1}=Y\left(J_{0}^{-1}u+Z_{2}+F\right)-\Lambda_{2}S-\hbar_{1}E_{1},\\ {\dot{Z}}_{2}=-\hbar_{2}\text{fal}\left(E_{1}\right), \end{array}$$

where *E*_1_ ∈ *R*^3×1^ means the ESO's estimation error, *Z*_1_, *Z*_2_ ∈ *R*^3×1^ denote the observer outputs, and *ℏ*_1_ and *ℏ*_1_ represent the observer gains. The function fal(·) is given by the following [17]:

(32) $$\begin{array}{c} \text{fal}\left(E_{1i}\right)=\left\{\begin{array}{cc} {\left|E_{1i}\right|}^{\gamma }\left(E_{1i}\right), & \left|E_{1i}\right|>\delta ,\\ \frac{E_{1i}}{\delta^{1-\gamma }}, & \left|E_{1i}\right|\leq \delta , \end{array}\right. \end{array}$$

where *i*=1,2,3, 0 < *γ* < 1, and *δ* > 0.

Define the observer error

(33) $$\begin{array}{c} E_{2}=D-Z_{2}. \end{array}$$

According to the analysis in [18], the observer error satisfies |*E*_2*i*_| ≤ *ζ*_*m*_,  *i*=1,2,3, where *ζ*_*m*_=max_*i*=1,2,3_{|*E*_2*i*_|} > 0.

### 4.2. Finite-Time Controller Design

Use (11) to approximate the nonlinear uncertainties (29).

(34) $$\begin{array}{c} F_{i}\left(x_{i}\right)=W_{i}^{*T}\phi_{1}\left(x_{i}\right)+\varepsilon_{i}, \end{array}$$

where $x_{i}\in {\left[e_{qi},{\dot{e}}_{qi},\omega^{r},{\dot{\omega }}^{r}\right]}^{T}\in R^{4}$ is the NN input vector, *W*^*∗*^ ∈ *R*^4^ represents the ideal weight vector, *ε*_*i*_ is the approximation error satisfying |*ε*_*i*_| ≤ *ε*_*N*_, *ε*_*N*_ > 0, and *ϕ*_1_(*x*) ∈ *R*^4^ denotes the Gaussian function (9).

An exponential reaching law is given by the following [19]:

(35) $$\begin{array}{c} \dot{S}=-\left(K_{1}S+K_{2}\cdot {\text{sig}}^{\gamma }\left(S\right)\right), \end{array}$$

where *K*_1_ > 0, *K*_2_ > 0, and 0 < *γ* < 1.

With the unknown nonlinear uncertainties *F* and the disturbances *D* estimated by the RBFNN and ESO, respectively, the finite-time control law *u* is given by

(36) $$\begin{array}{c} u=J_{0}\left(-K_{1}S-K_{2}{\text{sig}}^{\gamma }\left(S\right)-{\hat{W}}^{T}\phi_{1}\left(x\right)-Z_{2}-K_{3}YS\right), \end{array}$$

where *K*_3_ > 0, $\hat{W}=\text{diag}\left({\hat{W}}_{1},{\hat{W}}_{2},{\hat{W}}_{3}\right)$, and ${\hat{W}}_{i}$ is used to estimate ${\hat{W}}_{i}^{*}$ with *i*=1,2,3.

The update law of ${\hat{W}}_{i}$ is given by

(37) $$\begin{array}{c} {\dot{\hat{W}}}_{i}=\delta_{i}\left(Y_{i}S_{i}\phi_{1i}-\varpi_{i}{\hat{W}}_{i}\right), \end{array}$$

where *δ*_*i*_ > 0 and *ϖ*_*i*_ > 0 with *i*=1,2,3.

## 5. Stability Analysis

**Theorem 1 .**

Considering the tracking error system (8) and the control schemes (36) and (37), all the signals of the closed-loop system are UUB, and the sliding variable *S* and the tracking errors *e*_*q*_ and *e*_*ω*_ are FTUUB, respectively.

**Proof**

Design a Lyapunov function *V*_2_

(38) $$\begin{array}{c} V_{2}=\frac{1}{2}S^{T}S+\sum_{i=1}^{3}\frac{1}{2\delta_{i}}{\tilde{W}}_{i}^{T}{\tilde{W}}_{i}, \end{array}$$

where ${\tilde{W}}_{i}=W_{i}^{*}-{\hat{W}}_{i}$.

From (28), differentiating (38) leads to

(39) $$\begin{array}{c} {\dot{V}}_{2}=S^{T}\dot{S}-\sum_{i=1}^{3}\frac{1}{\delta_{i}}{\tilde{W}}_{i}^{T}{\dot{\hat{W}}}_{i}=S^{T}Y\left(J_{0}^{-1}u+F+D\right)-S^{T}\cdot \Lambda_{2}S-\sum_{i=1}^{3}\frac{1}{\delta_{i}}{\tilde{W}}_{i}^{T}{\dot{\hat{W}}}_{i}. \end{array}$$

Substituting (34) and (36) into (39), one has

(40) $$\begin{array}{c} {\dot{V}}_{2}=S^{T}Y\left(J_{0}^{-1}\cdot J_{0}\left(-K_{1}S-K_{2}{\text{sig}}^{\gamma }\left(S\right)-{\hat{W}}^{T}\phi_{1}-Z_{2}-K_{3}YS\right)+W^{*T}\phi_{1}+\varepsilon +D\right)\\ -\Lambda_{2}\sum_{i=1}^{3}S_{i}^{2}-\sum_{i=1}^{3}\frac{1}{\delta_{i}}{\tilde{W}}_{i}^{T}{\dot{\hat{W}}}_{i}\\ \leq S^{T}Y\left(-K_{1}S-K_{2}{\text{sig}}^{\gamma }\left(S\right)+{\tilde{W}}_{1}^{T}\phi_{1}+\varepsilon +D-Z_{2}-K_{3}YS\right)-\sum_{i=1}^{3}\frac{1}{\delta_{i}}{\tilde{W}}_{i}^{T}{\dot{\hat{W}}}_{i}, \end{array}$$

where *ε*=[*ε*_1_, *ε*_2_, *ε*_3_]^*T*^.

From (33), (40) is modified as

(41) $$\begin{array}{c} \begin{array}{c} {\dot{V}}_{2}=S^{T}Y\left(-K_{1}S-K_{2}{\text{sig}}^{\gamma }\left(S\right)+{\tilde{W}}_{1}^{T}\phi_{1}+\varepsilon +E_{2}-K_{3}YS\right)-\sum_{i=1}^{3}\frac{1}{\delta_{i}}{\tilde{W}}_{i}^{T}{\dot{\hat{W}}}_{i} \end{array}. \end{array}$$

Substituting (37) into (40) yields

(42) $$\begin{array}{c} {\dot{V}}_{2}\leq -K_{1}\sum_{i=1}^{3}Y_{i}S_{i}^{2}-K_{2}\sum_{i=1}^{3}Y_{i}{\left|S_{i}\right|}^{1+\gamma }-K_{3}\sum_{i=1}^{3}Y_{i}^{2}S_{i}^{2}+\varepsilon_{N}\sum_{i=1}^{3}\left|Y_{i}\right|\left|S_{i}\right|\\ +\zeta_{m}\sum_{i=1}^{3}\left|Y_{i}\right|\left|S_{i}\right|+\sum_{i=1}^{3}\varpi_{i}{\tilde{W}}_{i}^{T}{\hat{W}}_{i}\\ \leq -K_{3}^{\prime }\sum_{i=1}^{3}Y_{i}^{2}S_{i}^{2}-\sum_{i=1}^{3}{\left(\sqrt{K_{3}^{\prime \prime }}\left|Y_{i}\right|\left|S_{i}\right|-\frac{\varepsilon_{N}+\zeta_{m}}{2\sqrt{K_{3}^{\prime \prime }}}\right)}^{2}+\sum_{i=1}^{3}\varpi_{i}{\tilde{W}}_{i}^{T}{\hat{W}}_{i}\\ +\frac{3\varepsilon_{N}^{2}}{4K_{3}^{\prime \prime }}+\frac{3\zeta_{m}^{2}}{4K_{3}^{\prime \prime }}, \end{array}$$

where *K*_3_=*K*_3_′+*K*_3_^″^.

From Young's inequality, the following relationships hold:

(43) $$\begin{array}{c} \varpi_{i}{\tilde{W}}_{i}^{T}\hat{W}\leq \varpi_{i}{\tilde{W}}_{i}^{T}\left(W_{i}^{*}-{\tilde{W}}_{i}\right)\leq -\frac{\varpi_{i}}{2}{\left\|{\tilde{W}}_{i}\right\|}^{2}+\frac{\varpi_{i}}{2}{\left\|W_{i}^{*}\right\|}^{2}. \end{array}$$

Substituting (43) into (42) yields

(44) $$\begin{array}{c} {\dot{V}}_{2}\leq -K_{3}^{\prime }\sum_{i=1}^{3}Y_{i}^{2}S_{i}^{2}-\frac{\varpi_{i}}{2}{\left\|{\tilde{W}}_{i}\right\|}^{2}+\frac{\varpi_{i}}{2}{\left\|W_{i}^{*}\right\|}^{2}+\frac{3\varepsilon_{N}^{2}}{4K_{3}^{\prime \prime }}\leq -\mu V_{2}+\Phi_{1}, \end{array}$$

where *μ*=min{2*K*_3_′*Y*_*i*_^2^, *δ*_*i*_*ϖ*_*i*_} and Φ_1_=(*ϖ*_*i*_/2)‖*W*_*i*_^*∗*^‖^2^+(3*ε*_*N*_^2^/4*K*_3_^″^).

According to (38)–(44), one can conclude that *S*, ${\tilde{W}}_{1}$, ${\tilde{W}}_{2}$, and ${\tilde{W}}_{3}$ are UUB. From (20) and the bounded values *W*_1_^*∗*^, *W*_2_^*∗*^, and *W*_3_^*∗*^, the uniform ultimate boundedness of *e*_*q*_, *e*_*ω*_, ${\hat{W}}_{1}$, ${\hat{W}}_{2}$, and ${\hat{W}}_{3}$ is guaranteed, and thus *Y*_*i*_ is also UUB. Due to (8) and (36), ${\dot{e}}_{\omega }$ and *u* both are UUB. Since ‖*ϕ*_1_(*x*)‖ is bounded in (9), one can conclude $\left\|S^{T}Y{\tilde{W}}^{T}\phi_{1}\right\|\leq \eta_{1}$, ‖*S*^*T*^*Yε*‖ ≤ *η*_2_, and ‖*S*^*T*^*YE*_2_‖ ≤ *η*_3_, where *η*_1_, *η*_2_, and *η*_3_ are positive constants.

Then, design a Lyapunov function

(45) $$\begin{array}{c} V_{3}=\frac{1}{2}S^{T}S, \end{array}$$

and from (28), ${\dot{V}}_{3}$ is

(46) $$\begin{array}{c} {\dot{V}}_{3}=S^{T}\dot{S}=S^{T}Y\left(J_{0}^{-1}u+W^{*T}\phi +\varepsilon +D\right)-\Lambda_{2}\sum_{i=1}^{3}S_{i}^{2}\leq S^{T}Y\left(J_{0}^{-1}u+W^{*T}\phi +\varepsilon +D\right). \end{array}$$

Substituting (36) into (46) yields

(47) $$\begin{array}{c} {\dot{V}}_{3}\leq S^{T}Y\left(-K_{1}S-K_{2}{\text{sig}}^{\gamma }\left(S\right)+{\tilde{W}}^{T}\phi_{1}+\varepsilon +E_{2}-K_{3}YS\right)\\ \leq -K_{1}\sum_{i=1}^{3}Y_{i}S_{i}^{2}-K_{2}\sum_{i=1}^{3}Y_{i}{\left|S_{i}\right|}^{1+\gamma }-K_{3}\sum_{i=1}^{3}Y_{i}^{2}S_{i}^{2}+S^{T}Y{\tilde{W}}^{T}\phi_{1}\\ +S^{T}Y\varepsilon +S^{T}YE_{2}\leq -\rho_{1}V_{3}-\rho_{2}V_{3}^{1+\gamma /2}+\Phi_{2}, \end{array}$$

where *ρ*_1_=min{2*K*_1_*Y*_*i*_, 1}, *ρ*_2_=min{2^1+*γ*/2^*K*_2_*Y*_*i*_, 1}, and Φ_2_=*η*_1_+*η*_2_+*η*_3_.

Thus, (47) can be transformed into the following form:

(48) $$\begin{array}{c} {\dot{V}}_{3}\leq -\left(\rho_{1}-\frac{\Phi_{2}}{V_{3}}\right)V_{3}-\rho_{2}V_{3}^{1+\gamma /2}\text{ or }{\dot{V}}_{3}\leq -\rho_{1}V_{3}-\left(\rho_{2}-\frac{\Phi_{2}}{V_{3}^{1+\gamma /2}}\right)V_{3}^{1+\gamma /2}. \end{array}$$

Due to Lemma 2 and (48), *S* can converge into Δ_*S*_ satisfying

(49) $$\begin{array}{c} \Delta S=\min\left\{\frac{\Phi_{2}}{\rho_{1}},{\left(\frac{\Phi_{2}}{\rho_{2}}\right)}^{2/1+\gamma }\right\}, \end{array}$$

within a finite-time bounded by

(50) $$\begin{array}{c} T_{s}\leq \frac{1}{\rho_{1}\left(1-\left(1+\gamma /2\right)\right)}\ln\frac{\rho_{1}V_{3}^{1-\left(1+\gamma /2\right)}\left(S_{0}\right)+\rho_{2}}{\rho_{2}}, \end{array}$$

where *S*_0_ is the initial value of *S*.

From (14), one has

(51) $$\begin{array}{c} \left|S_{j}\right|=\left|\text{sig}\left(e_{q_{j}}\right)+\frac{\Lambda_{1}}{2-a}{\text{sig}}^{2-a}\left(e_{\omega_{j}}+\Lambda_{2}\text{sig}\left(e_{q_{j}}\right)\right)\right|=\eta_{j},\;\left|\eta_{j}\right|\leq \Delta S, \end{array}$$

where *j*=1,2,3.

The terms (Λ_1_/2 − *a*)sig^2−*a*^(*e*_*ω*_*j*__+Λ_2_sig(*e*_*q*_*j*__)) and sig(*e*_*qj*_) are both positive or negative. Considering only positive case and Lemma 3, the following relationship exists without loss of generality:

(52) $$\begin{array}{c} \frac{{\left|e_{\omega_{j}}+\Lambda_{2}\text{sig}\left(e_{q_{j}}\right)\right|}^{2-a}}{2-a}\geq \left|e_{\omega_{j}}+\Lambda_{2}\text{sig}\left(e_{q_{j}}\right)\right|+\frac{a-1}{2-a}. \end{array}$$

Multiplying Λ_1_ and adding sig(*e*_*q*_*j*__) on both sides of (52), it has

(53) $$\begin{array}{c} \text{sig}\left(e_{q_{j}}\right)+\frac{\Lambda_{1}{\left(e_{\omega_{j}}+\Lambda_{2}\text{sig}\left(e_{q_{j}}\right)\right)}^{2-a}}{2-a}\geq \text{sig}\left(e_{q_{j}}\right)+\Lambda_{1}\left(e_{\omega_{j}}+\Lambda_{2}\text{sig}\left(e_{q_{j}}\right)\right)+\frac{\Lambda_{1}\left(a-1\right)}{2-a}. \end{array}$$

Substituting (53) into (51) yields

(54) $$\begin{array}{c} \text{sig}\left(e_{q_{j}}\right)+\Lambda_{1}e_{\omega_{j}}+\Lambda_{1}\Lambda_{2}\text{sig}\left(e_{q_{j}}\right)\leq \Delta \bar{S}, \end{array}$$

where $\Delta \bar{S}=\Delta S+\left(\Lambda_{1}\left(1-a\right)/2-a\right)$.

From (54), the attitude tracking errors *e*_*q*_ and angular velocity *e*_*ω*_ are finite-time stable. Thus, *e*_*q*_ and *e*_*ω*_ converge into small regions:

(55) $$\begin{array}{c} \left|e_{q_{j}}\right|\leq \frac{\Delta \bar{S}}{1+\Lambda_{1}\Lambda_{2}},\\ \left|e_{\omega_{j}}\right|\leq \frac{2\Delta \bar{S}}{\Lambda_{1}}, \end{array}$$

within a finite-time, respectively.

From the above discussion, the convergence time *T* of closed-loop system states in (8) is bounded, which satisfies

(56) $$\begin{array}{c} T=T_{r}+T_{s}\leq \frac{1}{{\bar{\Lambda }}_{1}\left(1-\iota_{0}\right)}\text{ln}\frac{{\bar{\Lambda }}_{1}V_{1}^{1-\iota_{0}}\left(e_{q}\left(0\right)\right)+{\bar{\Lambda }}_{2}}{{\bar{\Lambda }}_{2}}\\ +\frac{1}{\rho_{1}\left(1-\left(1+\gamma /2\right)\right)}\text{ln}\frac{\rho_{1}V_{3}^{1-\left(1+\gamma /2\right)}\left(S_{0}\right)+\rho_{2}}{\rho_{2}}. \end{array}$$

Consequently, the sliding variable *S* and the tracking errors *e*_*q*_ and *e*_*ω*_ are FTUUB.

This completes the proof.

**Remark 2 .**

The convergence time is determined by the parameters ${\bar{\Lambda }}_{1}$, ${\bar{\Lambda }}_{2}$, *K*_1_, *K*_2_, and *ι*_0_. From (56), we can find that when the parameters ${\bar{\Lambda }}_{1}$, ${\bar{\Lambda }}_{2}$, *K*_1_, and *K*_2_ are selected to be larger, the convergence speed will become faster while it will cause some chattering issues. Thus, the choice of ${\bar{\Lambda }}_{1}$, ${\bar{\Lambda }}_{2}$, *K*_1_, and *K*_2_ should be set appropriately to keep a balance between convergence speed and chattering.

## 6. Simulations Results

In this section, numerical simulations are displayed to show the attitude tracking performance. To indicate the superiority of the designed control scheme, two different control schemes are given for comparison, i.e., SFTSM controller [20] and adaptive linear sliding mode (ALSM) controller [21].

To intuitively display the physical meaning of the reference attitude trajectories, the reference attitude quaternion [*q*_0_^*r*^, *q*_*v*1_^*r*^, *q*_*v*2_^*r*^, *q*_*v*3_^*r*^] is expressed as

(57) $$\begin{array}{c} \left[\begin{array}{c} q_{0}^{r}\\ q_{v1}^{r}\\ q_{v2}^{r}\\ q_{v3}^{r} \end{array}\right]=\left[\begin{array}{c} \cos\frac{\psi_{d}}{2}\cos\frac{\theta_{d}}{2}\cos\frac{\phi_{d}}{2}+\sin\frac{\psi_{d}}{2}\sin\frac{\theta_{d}}{2}\sin\frac{\phi_{d}}{2}\\ \cos\frac{\psi_{d}}{2}\cos\frac{\theta_{d}}{2}\sin\frac{\phi_{d}}{2}-\sin\frac{\psi_{d}}{2}\sin\frac{\theta_{d}}{2}\cos\frac{\phi_{d}}{2}\\ \cos\frac{\psi_{d}}{2}\sin\frac{\theta_{d}}{2}\cos\frac{\phi_{d}}{2}+\sin\frac{\psi_{d}}{2}\cos\frac{\theta_{d}}{2}\sin\frac{\phi_{d}}{2}\\ \sin\frac{\psi_{d}}{2}\cos\frac{\theta_{d}}{2}\cos\frac{\phi_{d}}{2}-\cos\frac{\psi_{d}}{2}\sin\frac{\theta_{d}}{2}\sin\frac{\phi_{d}}{2} \end{array}\right], \end{array}$$

where [*ϕ*_*d*_, *θ*_*d*_, *ψ*_*d*_] are the desired Euler angles.

The parameters in (8) are *J*_0_=diag([0.1, 0.1, 0.1]) kg/m^2^, *ω*(0)=[0,0,0]^*T*^, and Δ*J*=diag([1,1,2]) kg/m^2^, and the external disturbances are set as *ϕ*(0)=*θ*(0)=*ψ*(0)=0°, and *d*(*t*)=[0.5  sin(0.1*t*), 0.5 sin(0.1*t*), 0.5  cos(*t*)]^*T*^ N · m.

In SFTSM, the parameters in (14) are set as Λ_1_=0.1, Λ_2_=0.4, and *a*=5/7. The parameters in (36) are chosen as *K*_1_=0.5, *K*_2_=1.1, *K*_3_=4, and *γ*=0.1. The number of RBFNN nodes is 10. The corresponding parameters in (9) and adaptive update law (37) are chosen as *μ*_*i*_ ∈ (−2,2), *a*_*i*_=*π*, *δ*_*i*_=0.1, *ϖ*_*i*_=0.2, and $\hat{W}\left(0\right)={\left[0,0,0,0\right]}^{T}$.

In ALSM, the linear sliding variable *S* is given by

(58) $$\begin{array}{c} S=e_{\omega }+\Lambda_{0}e_{q}, \end{array}$$

where Λ_0_=7.5, and the controller is

(59) $$\begin{array}{c} u=J_{0}\left(\Lambda_{0}e_{\omega }+{\dot{\omega }}^{r}+{\hat{\theta }}_{0}\mathrm{sgn}\left(S\right)-\left(K_{1}S+K_{2}{\text{sig}}^{\gamma }\left(S\right)\right)\right), \end{array}$$

in which the updating law of ${\hat{\theta }}_{0}$ is given by

(60) $$\begin{array}{c} {\dot{\hat{\theta }}}_{0}=c_{0}\left(\left\|S\right\|-\varepsilon_{0}{\hat{\theta }}_{0}\right), \end{array}$$

where *c*_0_=1, and the other parameters in the ALSM are set the same as those of SFTSM.

To illustrate the better tracking performance and transient convergence performance in SFTSM, the fixed initial Euler angles are selected with *ϕ*_*d*_=*θ*_*d*_=*ψ*_*d*_=10° as the reference trajectories. Figures 3 and 4 show the time response of control inputs in SFTSM and ALSM, respectively. It is concluded that the maximum amplitude of the control input is 10 N · m. The comparative results of the Euler angle tracking performance are shown in Figures 5–7. From Figure 5, the convergence time of *ϕ* in SFTSM is 0.5 s, and the convergence time of *ϕ* in ALSM is 1.5 s. Due to the same analysis in Figures 6 and 7, SFTSM can achieve faster convergence rate and better transient performance of Euler angles than ALSM.

For the purpose of showing the superiority of SFTSM, the corresponding attitude quaternion tracking performance in ALSM is presented in Figures 8–11. The convergence time of SFTSM is faster almost 1 s than ALSM, which means SFTSM can realize the better transient performance than ALSM. Based on the mentioned analysis, quaternion-based tracking performance in SFTSM is still outperformed than ALSM. According to Figures 3–11, it is illustrated that SFTSM can guarantee faster convergence speed and better tracking performance in the QUAV's attitude tracking control.

## 7. Conclusion

In this study, a finite-time convergent RBFNN-based adaptive controller has been constructed to resolve a tracking problem of quadrotor UAVs. Firstly, a SFTSMS is proposed to realize the finite-time convergence of the tracking errors, which can directly avoid the potential singularity problem without requiring any piecewise continuous functions. Besides, an auxiliary function is proposed to purposely prevent the hidden singularity issue caused by the error-related matrix in the controller design. Then, a finite-time attitude controller is designed to guarantee that the system states were FTUUB. With the presented control scheme by RBFNN and ESO, prior knowledge about the unknown nonlinear uncertainties and external disturbances is not required. Finally, comparative simulations have shown the effectiveness of the designed control scheme.

## Figures and Tables

**Figure 1:** The schematic of quadrotor UAVs.

**Figure 2:** The structure of RBFNN.

**Figure 3:** Control input in SFTSM.

**Figure 4:** Control input in ALSM.

**Figure 5:** The tracking performance of *ϕ*.

**Figure 6:** The tracking performance of *θ*.

**Figure 7:** The tracking performance of *ψ*.

**Figure 8:** The tracking performance of *q*_0_.

**Figure 9:** The tracking performance of *q*_*v*1_.

**Figure 10:** The tracking performance of *q*_*v*2_.

**Figure 11:** The tracking performance of *q*_*v*3_.

## Data Availability

The data used to support the findings of the study are available from the corresponding author upon request.
